# Optimization of Markov Queuing Model in Hospital Bed Resource Allocation

**DOI:** 10.1155/2020/6630885

**Published:** 2020-12-08

**Authors:** Jingna Wu, Bo Chen, Danping Wu, Jianqiang Wang, Xiaodong Peng, Xia Xu

**Affiliations:** ^1^The Affiliated Changshu Hospital of Soochow University, Changshu, Jiangsu 215500, China; ^2^The Office of Medical and Health Association, Changshu, Jiangsu 215500, China

## Abstract

Bed resources are the platform in which most medical and health resources in the hospital play a role and carry the core functions of the health service system. How to improve the efficiency of the use of bed resources through scientific management measures and methods and ultimately achieve the optimization of overall health resources is the focus of hospital management teams. This paper analyzes the previous research models of knowledge related to queuing theory in medical services. From the perspective of the hospital and the patient, several indicators such as the average total number of people, the utilization rate of bed resources, the patient stop rate, and the patient average waiting time are defined to measure the performance of the triage queue calling model, which makes the patient queue more reasonable. According to the actual task requirements of a hospital, a Markov queuing strategy based on Markov service is proposed. A mathematical queuing model is constructed, and the process of solving steady-state probability based on Markov theory is analyzed. Through the comparative analysis of simulation experiments, the advantages and disadvantages of the service Markov queuing model and the applicable scope are obtained. Based on the theory of the queuing method, a queuing network model of bed resource allocation is established in principle. Experimental results show that the queuing strategy of bed resource allocation based on Markov optimization effectively improves resource utilization and patient satisfaction and can well meet the individual needs of different patients. It does not only provide specific optimization measures for the object of empirical research but also provides a reference for the development of hospital bed resource allocation in theory.

## 1. Introduction

Health resources, as a major component of the provision of medical services, are extremely limited. How to rationally allocate and efficiently use health resources has become an urgent problem in the field of hospital management. Beds are one of the important resources for in-hospital emergency integration. Considering that other conditions will also affect indicators, such as staffing or bed allocation, we assume that these conditions are the same. If a hospital increases beds, it will increase investment of idle waste; on the contrary, if we reduce beds, the waiting time will be too long, and the patient satisfaction will decline. With the continuous deepening of medical reform, the competition between hospitals becomes more and more fierce. Hospital managers must consider how to strike a balance between the two in order to improve service quality, maximize returns, maintain a competitive advantage, and take into account social benefits [1–3].

With the continuous advancement and implementation of healthcare reform, scientifically and reasonably shortening the average hospitalization day, optimizing bed utilization has become a core issue that hospital management is paying close attention to. In the current medical environment, major domestic hospitals are exploring management models suitable for their own development, including refined management, target management, clinical path management, day wards, medical prepayment systems, and pay-by-case systems [4–6]. Relevant scholars have explored the use of their beds, mainly using prospective cohort studies [7, 8]. The conclusions show that the regularity and uninterruptedness of patient consultations, physician transfers, and discharges of physician consultations can be maintained from Monday to Sunday, which can effectively improve bed utilization. The researchers elaborated on three aspects of patient waiting time and service utilization analysis, system design, and appointment system [9]. They summarized the research of different scholars on the queuing theory applied to the medical system and applied the research results to personal clinics, medical facilities, and regional medical systems. Relevant scholars use a hospital as an example to classify patients into critically ill patients, general patients, and patients without appointments [10–12]. They combined the knowledge of queuing theory to simulate the patient flow in the emergency room and analyzed the specific situation of the hospital. When evaluating bed utilization in US hospitals, researchers built a simulation model with Simscript 11.5, which takes into account a series of indicators such as patient diagnosis, admission classification, length of stay, type of bed, and gender [13, 14]. The macroinfluencing factors of bed utilization are mainly related to the hospital or the country's policies [15]. At the microscale, they involve how the beds are configured, how the patients are placed, and how patients are admitted to the hospital. Relevant scholars have investigated and evaluated bed utilization efficiency in a certain area in Canada [16, 17]. The study found that, of the 2007 patient study subjects, 14.2% of patients did not meet the admission criteria, and the total length of hospital stay was 14,194 days, of which 22.8% were unreasonable. The study evaluated the unreasonable length of hospital stay and found that 49.2% of the unreasonable time was related to the doctor's job [18]. Although the average length of stay in the region decreased from 5.7 days to 5.39 days in 4 years, the average length of stay in 10.5% of hospitals still exceeded national standards [19–21]. This study shows that improper use of beds can lead to inefficient hospital operations or reduced alternative services. Some scholars believe that the hospital bed size is a nonlinear structure, and its management assessment is affected by uncertain environmental changes [22, 23]. At present, the calculation of bed size is a simple and modeled calculation method [24].

In theory, the common queuing problem in hospitals has always been a hotspot for domestic and foreign experts and scholars. Queue theory and corresponding improved model have been widely used to solve this problem. This study enriches the theoretical optimization of queuing problems in hospital management and provides an analysis and decision-making method for improving the queuing theory of hospitals and improving the efficiency of medical services. Specifically, the technical contributions of this paper are summarized as follows.

First, from the perspective of the hospital and the patient, several indicators such as the average total number of people, the utilization rate of bed resources, the patient's stopping rate, and the patient's waiting time are defined to measure the advantages and disadvantages of the triage queue calling model so that the queue is more reasonable. According to the actual task requirements of a hospital, a Markov queuing strategy based on Markov service is proposed, a mathematical queuing model is constructed, and simulation experiments are performed on the queuing model. Through experimental comparison and analysis, the advantages and disadvantages and applicable scope of the service Markov queuing model in this paper are obtained.

Second, this paper carried out a simulation experiment of 132 units of time on the simulation system and obtained the simulation results. The dynamic queue time and queue length obtained by simulating the queuing generated when matching the experts in each department and the queuing generated in each clinic are analyzed to find the congestion point of the queuing network system. After the parameter setting of the congestion point is improved, the result is compared with the original parameter state.

The rest of this paper is arranged as follows.  Section 2 discusses related theories and methods. In Section 3, Markov's hospital bed queuing strategy is studied.  Section 4 gives the simulation results and analysis. Finally, Section 5 summarizes the full text.

## 2. Related Theories and Methods

### 2.1. Refined Management Theory of Hospital Bed Resources

Refined management is not only an important way for hospitals to carry out ordinary management activities but also an important foundation for improving the overall management level of hospitals. The implementation of this management form in hospitals can significantly optimize hospital service procedures and improve service levels and patient satisfaction, which is of great significance to hospital development.

The refined management of hospital human resources is a management activity that takes full advantage of human resources in order to better complete the various tasks of the hospital. As a reasonable development and allocation of human resources, fine management effectively uses the combination of scientific management system, laws, and methods and refines classification management, level correspondence, and organizational structure.

Refined management includes outpatient emergency management, first-aid management, and discharge management within the medical procedures. It rationally connects the management of the above links. At the same time, it promotes the management of hospital departments and considers the patient as the center based on medical safety. It focuses on the key points, strengthens management, and improves the efficiency of service process operations. The system architecture of the hospital information platform is shown in Figure 1.

### 2.2. Features of the Queuing System

The following six basic characteristics are usually used to describe the queuing system:

1. Patient arrival mode
2. The time interval for patients to arrive in the queuing system is deterministic or random. Most patients in the hospital queuing system arrive randomly. Common input processes include Poisson input, fixed-length input, and Erlang input. Among them, Poisson input is most widely used in queuing systems. If the patient arrival interval follows a negative exponential distribution, then the number of patients who arrive within a certain time interval obeys the Poisson distribution. At this time, the arrival rule of the patients arriving in the system is called Poisson arrival. This situation is also the focus of queue theory.
3. Service model
4. Patient service hours are deterministic or random, and most service hours are random. The time rule of patients receiving services is often described by probability distribution. Generally, the probability distributions of random service hours are fixed-length distribution, negative exponential distribution, Erlang distribution, and so on. The service time of the queuing system usually follows a negative exponential distribution; that is, the time for each patient to receive the service is independently and identically distributed, and its distribution function is

(1) $$\begin{array}{c} B\left(t\right)=1-e^{-ut}\;\left(t\geq 0\right), \end{array}$$

  where *u* > 0 is a constant, representative of the average service rate per unit time, and 1/*u* is the average service time. Service methods are divided into single or batch.
(3) Queuing rules
  The most common queuing rules are first-come-first-served services, such as medical appointments and queuing for medication. Under the first-come-first-served service rule, patients receive services in the order of arrival. General service systems use this queuing rule. Other queuing rules include first-come-first-served, nonpreemptive priority, and preemptive priority. First-come-first-served services include hospitals for emergency patients. Preemptive priority means that when a patient with higher priority arrives at the system, the patient who is receiving the service must stop the service and be replaced to serve such patients, like the hospital emergency room for critically ill patients. Nonpreemptive priority means that when a higher priority patient arrives at the service system, the patient who is receiving the service must wait for the service to be completed before receiving the service, such as a care number.
(4) Serviceability
  Generally, the queuing system has a queuing upper limit. When the queuing upper limit is exceeded, the patients who arrive will be rejected, which is a loss system. There is no upper limit for waiting. The hybrid system is a queuing service rule that combines the loss system and the waiting system. There are both waiting and loss situations. For example, the patient decides to stay in consideration of the length of the queue and the length of the waiting time. There are two main types of mixed systems. One is the limitation of the length of the team; that is, when the number of patients waiting in line for service exceeds the prescribed number, the subsequent patients automatically leave. The second is the limited waiting time; that is, when patients wait in line for more than a certain time, they will automatically leave.
(5) Number of bed resources
  The main attribute of the service window is the number of bed resources, and its type is a single bed resource or multiple bed resources. If it is a multibed resource system, it can be divided into three types: parallel system, series system, and hybrid type. The most basic type is the parallel multibed resource. There are many queuing situations in the hospital's queuing network.
(6) Service stage
  A service system is usually a service phase or multiple service phases. The treatment of patients in hospitals often needs to go through multiple service stages, such as outpatient visits; usually, it needs to go through multiple service stages such as registration service stage, consultation service stage, payment service stage, inspection service stage, and return-to-treatment and medication collection. The schematic diagram of the hospital triage system is shown in Figure 2.

### 2.3. Markov Model Analysis

According to the characteristics of the probability distribution, from one state to another state in the Markov chain, it can also maintain the current state. The random change between states is called transition, and the probability of changing between different states is called transition probability. The Markov chains *X*_1_, *X*_2_, *X*_3_,… describe a state time series, where each state value is related to a limited number of states before the current state. The Markov chain reflects a series of variables with Markov properties. The set of all possible values is the range of the variable, which is the state space, and the value of *X*_*n*_ represents the state at time *n*.

A Markov chain can be represented by a probability distribution. The probability distribution *P*(*X*_*n*+1_=*X*_*n*_) is called the “one-step transition probability” in a random process. The multistep transition probability can be derived from the one-step transition probability; that is,

(2) $$\begin{array}{c} P\left(X_{n+2}|X_{n}\right)=\int P\left(X_{n+2},X_{n+1}|X_{n}\right)\text{d}X_{n+1}. \end{array}$$

Markov process is a typical stochastic process, which is applicable to both interval and time series. This theory is mainly to study the state and transition of sequences. Markov model is a prediction method that performs random analysis on time series. The Markov model is a prediction method that predicts whether an object may be in a certain state in the future according to the initial probability of different objects in different states and the transition probability between different states.

## 3. Hospital Bed Queuing Strategy Based on Markov

### 3.1. Steps to Build a System Transition Probability Matrix

For multidimensional state space, it will be more complicated if you use manual calculation. The classic matrix geometry algorithm is more suitable for solving two-dimensional state space. For 3D state space, other methods need to be found for solving. In this paper, a computer-based method is used to solve the transition probability matrix of a multidimensional Markov chain. The steps are as follows.

 
*Step 1*. We sort all the multidimensional state spaces with a dictionary sorting method and study the form of the state.
 
*Step 2*. We define a functioning state (*p*) to describe the *p*^th^ element in the sorted state space. In the proposed Markov model, the way the state is formed is very important; it has a great influence on the constructor state (*p*). Different formation methods will produce different functions. However, we find that, in most multidimensional Markov models, the state space is formed layer by layer. Therefore, state (*p*) will be constructed in the following way.
 
*Step 3*. We construct the transition probability function transition (*n*, *A*) between states *A* and *B*. Because the transition situation designed in this paper is more complicated, the transition probability should be determined according to the specific problem.
 
*Step 4*. We obtain the state transition matrix *Q* according to the transition probability between states.

### 3.2. Experimental Design

#### 3.2.1. Definition and Solution of the Queuing Model

Assume that there are two bed resources *S*1 and *S*2 in the system, where *S*1 serves C1 patients, the patients arrive at *λ*_1_, the service rate is *u*1, and the formed team length is *n*_1_; *S*2 serves *C*2 patients, the patients arrive at *λ*_2_, the service rate is *u*2, and the length of the formed team is *n*_2_, of which *λ*_1_ > *λ*_2_. When *n*_1_ = *F*_1_, *C*1 patients leave the queuing system; when *n*_2_ = *F*_2_, *C*2 patients leave the queuing system, where *F*_1_ > *F*_2_.

*(1) State Space*. We define *n*_1_ (*t*) as the total queue length of *S*1 bed resources and *n*_2_ (*t*) as the total queue length of *S*2 bed resources, and then each instantaneous state space can be expressed as

(3) $$\begin{array}{c} X_{t}=\left[n_{1}\left(t\right),n_{2}\left(t\right)\right], \end{array}$$

where *n*_1_ (*t*) represents the total queue length of bed resource *S*1 at time *t* and *n*_2_ (*t*) represents the total queue length of bed resource *S*2 at time *t*.

*(2) Transfer Process*. The transition relationship between all states in the state space obeys the continuous Markov process. Predecessors have studied the laws that such a transition process meets. The birth and death process of the system is given in the following. According to Markov theory, the system transition probability is

(4) $$\begin{array}{c} q=\left\{\begin{array}{cc} \lambda_{1} & \left(n_{1},n_{2}\right)⟶\left(n_{1}+1,n_{2}\right)\\ u_{1} & \left(n_{1},n_{2}\right)⟶\left(n_{1}-2,n_{2}\right)\\ \lambda_{2} & \left(n_{1},n_{2}\right)⟶\left(n_{1},n_{2}+1\right)\\ u_{2} & \left(n_{1},n_{2}\right)⟶\left(n_{1},n_{2}-2\right). \end{array}\right. \end{array}$$

According to the transition probability between states, a state transition matrix *Q* is obtained.

#### 3.2.2. Performance of the Queuing Model

Using steady-state probability and transition probability matrix, we can obtain the following performance characteristics.

*(1) The Average Total Number of People in the System*. When the system is in a steady state, the total number of people in each state in the state space is multiplied by the steady-state probability of the state, and the summed value is the average total number of people in the system:

(5) $$\begin{array}{c} E\left(S\;:F_{1}\;:F_{2}\right)=\sum_{n_{1}=0}^{F_{1}}\sum_{n_{2}=0}^{F_{2}}\left(n_{1}+n_{2}\right)\pi \left(n_{1},n_{2}\right). \end{array}$$

*(2) The Average Number of People Waiting in the System*. When the system is in a steady state, the value of the waiting number can be computed using the total number of people minus the number of patients receiving services, and the value multiplied by the steady-state probability is the system's average waiting number.

(6) $$\begin{array}{c} E\left(Q\;:F_{1}\;:F_{2}\right)=\sum_{n_{1}=0}^{F_{1}}\sum_{n_{2}=0}^{F_{2}}\left(n_{1}+n_{2}-1\right)\left[\pi \left(n_{1},n_{2}\right)|n_{1}n_{2}=0\right]. \end{array}$$

*(3) Resource Utilization Rate of Each Bed*. According to the definition of steady-state probability, that is, the probability that the system is in various states after an infinite time tends to stabilize, this probability also includes the meaning of the time component in each state. Therefore, the probability that each bed resource is busy during steady state is equal to their respective utilization rates. Therefore, the utilization rate of each bed resource can be obtained as follows.

The utilization rate of bed resource is *S*1, that is, the probability that *S*1 is in a busy period when *S*1 reaches steady state. The probability when there is always a patient in cohort *n*_1_ is

(7) $$\begin{array}{c} \rho_{s_{1}}=\sum_{n_{1}=0}^{F_{1}}\sum_{n_{2}=0}^{F_{2}}\left[\pi \left(n_{1},n_{2}\right)|n_{1}\neq 0\right]. \end{array}$$

The utilization rate of bed resource is *S*2, that is, the probability that *S*2 will be busy when *S*2 reaches steady state. The probability that patients in the *n*_2_ cohort will always exist is

(8) $$\begin{array}{c} \rho_{s_{2}}=\sum_{n_{1}=0}^{F_{1}}\sum_{n_{2}=0}^{F_{2}}\left[\pi \left(n_{1},n_{2}\right)|n_{2}\neq 0\right]. \end{array}$$

*(4) Patient Waiting Time in the System*. Patient waiting time is the average time that all patients wait for service in the system under steady-state conditions. When the system is in a steady state, the waiting time for a patient is the number of all patients in front of it multiplied by the time required for a single patient to receive service. Among them, the time required for a single patient to receive service is 1/*u*. If there is only one patient receiving service in a certain state, the waiting time is 1/*u*. If there are *i* patients before, the waiting time is (*i* − 1)/*u*. Then the waiting time in each state is multiplied by its steady-state probability and summed, which is the average waiting time of the patient in the system.

The waiting time for the *C*1 patient in the system is

(9) $$\begin{array}{c} E_{c_{1}}\left(W\;:F_{1}\;:F_{2}\right)=\sum_{n_{1}=0}^{F_{1}}\sum_{n_{2}=0}^{F_{2}}\left[\frac{n_{1}}{u_{1}}\pi \left(n_{1},n_{2}\right)\right]. \end{array}$$

The waiting time for *C*2 patients in the system is

(10) $$\begin{array}{c} E_{c_{2}}\left(W:F_{1}:F_{2}\right)=\sum_{n_{1}=0}^{F_{1}}\sum_{n_{2}=0}^{F_{2}}\left[\frac{n_{2}}{u_{2}}\pi \left(n_{1},n_{2}\right)\right]. \end{array}$$

The total patient waiting time in the system is the average of the waiting time of the *C*1 patient in the system and the waiting time of the *C*2 patient in the system, as shown in the following formula:

(11) $$\begin{array}{c} E\left(W\;:F_{1}\;:F_{2}\right)=0.5\cdot \left(E_{c_{1}}+E_{c_{2}}\right). \end{array}$$

### 3.3. Results Analysis

#### 3.3.1. Average Total Number of People

From Table 1, it can be seen that the total number of people in both queuing systems increases with the increase of *F*_1_. This shows that the higher the tolerance of *C*1 patients, the more crowded the system, and the more waiting people in the system measure the advantages and disadvantages. At the same time, it can be seen in the table that the change gradually slows down, indicating that the increase in the number of people tends to moderate with the increase of *F*_1_. This shows that the system itself is buffered against tolerance changes. At the same time, the number of people that the system can accept is also limited. When the patient's impatience reaches a certain level, the number of people in the system will reach the limit and no longer increase.

In addition, it can be seen from the table that the number of waiting people in the queuing system using the sharing strategy is smaller than that in the queuing system that does not adopt this strategy, and the difference between the two becomes larger and larger as *F*_1_ increases. This is because when the tolerance limit of *C*1 patients becomes larger, more patients will enter the *S*1 system and wait for services. The queuing system using the sharing strategy can effectively divert *C*1 patients who are waiting to receive services. Some *C*1 patients can enter the *S*2 bed resource to receive services and leave the system. Therefore, the waiting number of the queuing systems using the sharing strategy is smaller than that of the ordinary system. At the same time, as the patient's tolerance changes, *F*_1_ increases, which will cause more *C*1 patients to enter the system to wait for services, and the waiting number of nonshared systems will continue to rise. After adopting the sharing strategy, because the arrival rate of *C*2 patients is relatively low, more *C*1 patients can use the *S*2 bed resources to complete the service and leave the system. Therefore, as *F*_1_ increases, the gap between the two systems continues to grow.

#### 3.3.2. Bed Resource Utilization

Comparing the utilization of *S*1 bed resources, it can be seen from Table 2 that, for *S*1 bed resources, the utilization rate of the system using the sharing strategy is lower than that of the system not using the sharing system. This is because, after adopting the sharing strategy, some *C*1 patients will enter the *S*2 bed resources to receive services, thus resulting in lower utilization of the *S*1 bed resources.

For comparison of *S*2 bed resource utilization, from the analysis of *S*1 bed resource utilization analysis, it can be concluded that, after the sharing strategy is adopted, some *C*1 patients enter *S*2 bed resources to receive services, which will inevitably lead to the improvement of *S*2 bed resource utilization. As shown in Table 3, it can be seen from the table that the utilization of *S*2 bed resources has improved significantly.

#### 3.3.3. Probability of Patient Stopping

Table 4 shows the change of the stopping probability of different patients in the two-system model to the tolerance limit of *C*1 patients. It can be seen in the table that the increase of the tolerance limit of *C*1 patients is very effective in reducing the probability of stopping. As the patient's tolerance limit increases, the probability of stopping is greatly reduced. From the perspective of system analysis, the stopping probability of *C*1 patients in the sharing system is significantly lower than that of the ordinary model. This is because the sharing strategy has a significant shunt effect on *C*1 patients, which makes more patients enter the system to receive services. But the stopping probability of *C*2 patients is not sensitive to changes in the tolerance limit of *C*1 patients. The reason is that, in the general model, *C*1 patients do not have any effect on *C*2 patients, so the stopping probability of *C*2 patients does not change. However, in the sharing system, because *C*1 patients will enter the *S*2 cohort to receive services, affecting some *C*2 patients, they will not be able to enter the system to receive services, resulting in a higher probability of stopping. Therefore, we can see that the stopping probability of *C*2 patients in the sharing system is higher than that of the ordinary system. But its own changes are not sensitive to the tolerance limit of *C*1 patients.

#### 3.3.4. Patient Waiting Time

Table 5 shows the comparison of waiting time for *C*1 patients in the two queuing system models. It can be clearly seen from the table that, as the tolerance limit of *C*1 patients increases, their waiting time also shows an upward trend. However, in the system without the sharing strategy, the waiting time of *C*1 patients increased faster and significantly higher than the system with the sharing strategy, while the waiting time of the sharing strategy system did not change much and was at a low level. This is because in the ordinary system, as the tolerance endurance of *C*1 patients increases, more and more *C*1 patients enter the *S*1 queue waiting to receive services, so their waiting time continues to increase. After adopting the sharing strategy, because some *C*1 patients entering the *S*1 queue can be transferred to the *S*2 queue to receive services, there is no need to wait too long to get services to leave the system. Therefore, the waiting time of *C*1 patients in the sharing system is lower than that of the ordinary system, and it can be seen that the sharing strategy has a significant effect on reducing the waiting time of *C*1 patients.

Table 6 shows a comparison of waiting times for *C*2 patients. First, it can be seen from the table that the waiting time of *C*2 patients in both systems is relatively stable, indicating that the tolerance limit of *C*1 patients has little effect on the waiting time of *C*2 patients. The waiting time in the system model using the sharing strategy is higher than the ordinary model without this strategy. This is because some *C*1 patients enter the *S*2 cohort to receive services in the system model of the sharing strategy, thus increasing the waiting time of some *C*2 patients. Judging from the waiting time of *C*2 patients alone, the split strategy system model has no advantage. But because the queuing system designed in this paper contains two bed resources and has two queues and two types of patients, it is necessary to consider the advantages and disadvantages of this queuing strategy from the perspective of the system as a whole.

Table 7 shows the overall patient waiting time in both types of systems. The total patient waiting time is the sum of the waiting time of the *C*1 patient and the waiting time of the *C*2 patient in the system. It can be seen from the table that the overall waiting time of patients in the common model without the sharing strategy is higher than that of the system model with the sharing strategy. And with the increase of the tolerance limit of *C*1 patients, the waiting time of patients under the common system model also increases rapidly, and the gap between the system models after adopting the sharing strategy is increasing. Therefore, from the perspective of the overall waiting time of patients in the system, the queuing system model using the sharing strategy is better than the ordinary model, and the greater the tolerance limit of *C*1 patients, the more obvious the effect.

## 4. Simulation Results and Analysis

### 4.1. Queuing System Optimization

The purpose of establishing a queuing model is to obtain the optimal parameter combination by changing the service parameters and measuring the service cost and the waiting cost in order to obtain the length and duration of the queuing team under the steady state of the system. In the bed resource allocation queuing system in this paper, the purpose of optimization is to obtain the best combination of the number of experts *r* in each department and the number of bed resource allocations *s*.

We take *z* as the average of the total cost per unit time in a steady state:

(12) $$\begin{array}{c} z=c_{s}^{\prime }s+c_{w}L. \end{array}$$

Among them, *c*_*s*_′ is the service cost for each bed resource unit time, *c*_*w*_ is the cost of each patient staying in the system, *s* is the number of bed resource allocations, and *L* is the average queue length. We think of *z* as a function of *s*, write *z* = *z* (*s*), and find *s*^*∗*^ that minimizes *z* (*s*).

Because *s* can only take integers and *z* (*s*) is not a continuous function, it cannot be calculated by calculus. According to the characteristic that *z* (*s*^*∗*^) should be the smallest, we get

(13) $$\begin{array}{c} \left\{\begin{array}{c} z\left(s^{*}\right)<z\left(s^{*}-1\right),\\ z\left(s^{*}\right)<z\left(s^{*}+1\right). \end{array}\right. \end{array}$$

We bring *z* into the above formula and simplify it:

(14) $$\begin{array}{c} L\left(s^{*}\right)-L\left(s^{*}+1\right)<\frac{c_{s}^{\prime }}{c_{w}}<L\left(s^{*}-1\right)-L\left(s^{*}\right). \end{array}$$

We solve the value of *L* when *r* = 1, 2, 3,…, and *s* = 1, 2, 3,…, in turn, and calculate the difference between two adjacent *L* values. Since *cs*′/*cw* is a known number, the optimal *s*^*∗*^ can be obtained according to which inequality related to *s* falls.

### 4.2. Simulation Results

Because the hospital's application for the allocation of bed resources is completed during working hours, it is assumed that 6 hours of the day can be applied for the allocation of bed resources at the basic level hospitals, 22 working days per month and 132 hours per month. Based on the previous parameters set, this paper simulates 132 units of time for a one-month bed resource allocation queuing system. In the end, 2224 cases of bed resource allocation applications were generated, and 1,716 cases were completed. The service rate of bed resource allocation applications reached 79.9%.

### 4.3. Analysis of Queuing Results

In order to allow the system to configure the applicant service for more bed resources, the performance of the system can be tested by adjusting parameters. Through the above analysis, in order to improve the system's pass rate, the congestion problem of the Department of Internal Medicine is mainly needed to be solved. The main cause of the congestion is that the probability of primary medical departments applying for the Department of Internal Medicine is very high, accounting for 53.46% of the total application, the preset Department of Internal Medicine has 14 experts, and the number is small, so it is envisaged that the number of experts in the Department of Internal Medicine can be increased to reduce the queue length and duration and improve the service rate of the entire queuing system.

Because the parameter combinations of the entire system are related to each other, if you want to comprehensively analyze the impact of each parameter on the entire queuing system, you need to obtain a 7-dimensional array, that is, the parameters of the 3 medical departments, the number of consultation rooms, and the length and duration of the queuing team. It is also not easy to analyze. It can be seen from the preset queuing system of the clinic that only the Department of Internal Medicine has the greatest influence on the entire queuing system. Therefore, this paper only conducts an experimental analysis of the combination of parameters of the number of experts and the number of clinics in the Department of Internal Medicine. On the premise that all other parameters are unchanged, by adjusting the number of experts in the Department of Internal Medicine, under the condition of different numbers of clinics, the queuing time and the queue length of the Department of Internal Medicine of each queuing system are simulated. We get the data in Table 8.

The number of experts in the medical department does affect the length and duration of the queue. When the number of consultation rooms is insufficient, the length and duration of the queue can be appropriately reduced. However, when the number of consultation rooms is sufficient, it has little effect on the queuing system. On the whole, the number of experts in the medical department has a limited impact on the queue length and waiting time of the system.

The medical resource allocation of bed resources mentioned in this paper mainly refers to consultation rooms and experts. General resource allocation optimization considers the cost of input resources and the benefits generated by the system from an economic perspective. However, the allocation of bed resources is a key project supported by the state, and the social benefits generated cannot be simply measured from an economic perspective. Therefore, this paper only optimizes the queuing system from the perspective of improving service efficiency.

## 5. Conclusion

This paper analyzes the previous research models of related knowledge of queuing theory in medical services and summarizes the advantages and disadvantages of the queuing model so that it can be used as a constraint in the subsequent queuing optimization model. From the perspective of the hospital and the patient, several indicators such as the average total number of people, the utilization rate of bed resources, the patient stop rate, and the patient waiting time are defined to measure the advantages and disadvantages of the triage queue calling model, which makes the patient queue more reasonable. According to the actual task requirements of a hospital, a Markov queuing strategy based on Markov service is proposed. A mathematical queuing model is constructed, the process of solving the steady-state probability based on Markov theory is analyzed, and a simulation experiment is performed on the queuing model. Through experimental comparison and analysis, the advantages and disadvantages and applicable scope of the service Markov queuing model in this paper are obtained. This paper proposes the use of queuing theory to model and analyze the allocation of bed resources and uses simulation to obtain a dynamic waiting time length and waiting time change chart, which avoids that the theoretical derivation cannot be closer to the actual situation and also avoids cumbersome operations when solving related quantitative indicators. According to the parameters, the queuing system is simulated, and the dynamic queuing time length and queuing time map during the allocation of bed resources are found. It is found that the internal medical queuing is relatively congested. By analyzing the number of consultation rooms and the experts of the Department of Internal Medicine, the influence of the queuing team length and time is obtained. It comes to the conclusion that experts in the Department of Internal Medicine do not need much change. Based on the time-series prediction of the bed resource allocation based on the bed resource allocation data, the approximate bed resource allocation in the next few months is obtained. The bed resource allocation queuing model established in this paper can still be applied well. In the future, some advanced machine learning technologies can be used to further improve the performance of the bed resource allocation queuing model.

## Figures and Tables

**Figure 1:** The system architecture of the hospital information platform.

**Figure 2:** Schematic diagram of the hospital triage system.

**Table 1:** Change of the average patient number of the system with *F*_1_.

Models	*F*_1_ score					
	5	10	15	20	25	30
Markov queuing model	3	4.5	5	5.2	5.7	6.3
Ordinary queuing model	2.8	4.3	4.6	4.7	5.1	5.2

**Table 2:** Change of resource utilization of *S*1 beds with *F*_1_.

Models	*F*_1_ score					
	5	10	15	20	25	30
Markov queuing model	0.65	0.67	0.68	0.74	0.76	0.86
Ordinary queuing model	0.62	0.63	0.64	0.68	0.69	0.76

**Table 3:** Change of resource utilization of *S*2 beds with *F*_1_.

Models	*F*_1_ score					
	5	10	15	20	25	30
Markov queuing model	0.52	0.53	0.54	0.56	0.59	0.62
Ordinary queuing model	0.38	0.41	0.43	0.44	0.45	0.46

**Table 4:** Variation of patient's stopping probability with *F*_1_.

Models	*F*_1_ score					
	5	10	15	20	25	30
Markov queuing model with *C*1	0.21	0.19	0.16	0.15	0.12	0.09
Markov queuing model with *C*2	0.03	0.03	0.03	0.03	0.03	0.03
Ordinary queuing model with *C*1	0.1	0.07	0.06	0.05	0.04	0.01
Ordinary queuing model with *C*2	0.01	0.01	0.01	0.01	0.01	0.01

**Table 5:** *C*1 patient waiting time as a function of *F*_1_.

Models	*F*_1_ score					
	5	10	15	20	25	30
Markov queuing model	0.8	0.9	1	1.1	1.2	1.3
Ordinary queuing model	1.8	2.2	3.1	4	4.9	5.1

**Table 6:** *C*2 patient waiting time as a function of *F*_1_.

Models	*F*_1_ score					
	5	10	15	20	25	30
Markov queuing model	1.2	1.25	1.25	1.31	1.33	1.35
Ordinary queuing model	0.5	0.53	0.62	0.75	0.8	0.9

**Table 7:** Patient overall waiting time with *F*_1_.

Models	*F*_1_ score					
	5	10	15	20	25	30
Markov queuing model	0.9	0.9	1	1.1	1.2	1.3
Ordinary queuing model	1.4	1.7	2.4	2.7	3.2	3.5

**Table 8:** Length and duration of the queuing team under the parameters of the number of experts and the number of consultation rooms in the Department of Internal Medicine.

Office 1	Number of experts	8	9	10	11	12	13	14
	Queue time	35	36	32	34	33	37	38
	Queue length	10	8	8	7	9	12	11
	Number of experts	15	16	17	18	19	20	21
	Queue time	30	24	22	21	25	22	23
	Queue length	8	8	12	11	7	6	3

Office 2	Number of experts	8	9	10	11	12	13	14
	Queue time	19	20	22	21	23	24	24
	Queue length	4	5	5	6	9	5	11
	Number of experts	15	16	17	18	19	20	21
	Queue time	17	18	18	16	19	21	24
	Queue length	12	7	7	6	10	11	9

Office 3	Number of experts	8	9	10	11	12	13	14
	Queue time	9	7	4	12	8	11	10
	Queue length	9	10	7	6	6	12	9
	Number of experts	15	16	17	18	19	20	21
	Queue time	9	8	7	7	13	16	21
	Queue length	6	5	7	11	10	7	4

## Data Availability

The labeled dataset used to support the findings of this study are available from the corresponding author upon request.
